RETRACTED

# l-Arginine Uptake by Cationic Amino Acid Transporter Promotes Intra-Macrophage Survival of *Leishmania donovani* by Enhancing Arginase-Mediated Polyamine Synthesis

**DOI:** 10.3389/fimmu.2017.00839

**Published:** 2017-07-26

**Authors:** Abhishek Mandal, Sushmita Das, Ajay Kumar, Saptarshi Roy, Sudha Verma, Ayan Kumar Ghosh, Ruby Singh, Kumar Abhishek, Savita Saini, Abul Hasan Sardar, Bidyut Purkait, Ashish Kumar, Chitra Mandal, Pradeep Das

**Affiliations:** ^1^Department of Molecular Biology, Rajendra Memorial Research Institute of Medical Sciences (ICMR), Patna, India; ^2^Department of Microbiology, All India Institute of Medical Sciences (AIIMS), Patna, India; ^3^Cancer Biology and Inflammatory Disorder Division, CSIR-Indian Institute of Chemical Biology, Kolkata, India; ^4^Department of Biotechnology, National Institute of Pharmaceutical Education and Research, Hajipur, India

**Keywords:** macrophage, *Leishmania*, l-arginine, CAT-2, arginase, nitric oxide, polyamine, cytokine

## Abstract

The survival of intracellular protozoan parasite, *Leishmania donovani*, the causative agent of Indian visceral leishmaniasis (VL), depends on the activation status of macrophages. l-Arginine, a semi-essential amino acid plays a crucial regulatory role for activation of macrophages. However, the role of l-arginine transport in VL still remains elusive. In this study, we demonstrated that intra-macrophage survival of *L. donovani* depends on the availability of extracellular l-arginine. Infection of THP-1-derived macrophage/human monocyte-derived macrophage (hMDM) with *Leishmania*, resulted in upregulation of l-arginine transport. While investigating the involvement of the transporters, we observed that *Leishmania* survival was greatly impaired when the transporters were blocked either using inhibitor or siRNA-mediated downregulation. CAT-2 was found to be the main isoform associated with l-arginine transport in *L. donovani*-infected macrophages. l-arginine availability and its transport regulated the host arginase in *Leishmania* infection. Arginase and inducible nitric oxide synthase (iNOS) expression were reciprocally regulated when assayed using specific inhibitors and siRNA-mediated downregulation. Interestingly, induction of iNOS expression and nitric oxide production were observed in case of inhibition of arginase in infected macrophages. Furthermore, inhibition of l-arginine transport as well as arginase resulted in decreased polyamine production, limiting parasite survival inside macrophages. l-arginine availability and transport regulated Th1/Th2 cytokine levels in case of *Leishmania* infection. Upregulation of l-arginine transport, induction of host arginase, and enhanced polyamine production were correlated with increased level of IL-10 and decreased level of IL-12 and TNF-α in *L. donovani*-infected macrophages. Our findings provide clear evidence for targeting the metabolism of l-arginine and l-arginine-metabolizing enzymes as an important therapeutic and prophylactic strategy to treat VL.

RETRACTED

## Introduction

*Leishmania donovani*, the causative agent of Indian visceral leishmaniasis (VL) exhibit a dimorphic life cycle, transmitted by a *Phlebotomine* sand fly vector as flagellated promastigotes and inhabit within mammalian macrophages (MΦs) as amastigotes. The destiny of intracellular amastigotes relies predominantly on the MΦ-activation status, which is largely affected by different cytokines and chemokines (1–3).

While diverse molecules and characteristics of macrophages are reciprocally or mutually exclusively related to the activation status of macrophages, the dichotomous regulation of l-arginine metabolism is at the center of the different functions that are associated with classically or alternatively activated macrophages. Classically activated MΦs can generate anti-microbicidal molecules and oxidative mediators and eliminate parasites successfully, whereas “alternatively” activated MΦs augment parasite persistence (4, 5). Although two apparent types of MΦ activation can lead to antithetical outcomes of infection, these two pathways employ l-arginine as a common substrate for their enzymatic activities.

l-Arginine is a non-essential amino acid for healthy adult human, but it has to be supplemented during growth or various disease states (6, 7) and has thus been characterized as a semi- or conditionally essential amino acid. Mammalian l-arginine metabolism is critical both at the level of the whole organism (6, 7) and at the level of the discrete cell types (8). In macrophages, l-arginine is an antecedent for principally two crucial metabolic pathways: it is metabolized either by inducible nitric oxide synthase (iNOS) to nitric oxide (NO) and citrulline or it is hydrolyzed by arginase to ornithine and urea. Arginase has two isoforms (arginase 1 and arginase 2), which catalyze the alike biochemical reaction but vary in cellular expression, cell-type-specific regulation, and subcellular localization one being cytosolic and the other mitochondrial, respectively (9, 10). The availability of l-arginine regulates the expression of different genes (7) and it is reported that l-arginine from the extracellular milieu is vital for iNOS-mediated NO production (11, 12). Furthermore, it is documented that the extent of arginase activities are indicators of disease extremity in human VL and in HIV infections (13–15).

RETRACTED

Ornithine, the downstream molecule of l-arginine metabolism, is metabolized by ornithine decarboxylase, a rate-limiting enzyme, to produce polyamines which regulate several cellular processes like DNA replication, protein translation, cellular growth, and differentiation (16, 17). It is reported that polyamines enhance the growth of intracellular *Leishmania* amastigotes inside murine macrophages (18) and arginase-expressing granulocytes (13, 14). However, little is known about the role of polyamines in immune regulation. Therefore, macrophage l-arginine metabolism may have wide ranging implications for the type and outcome of immune responses.

Importance of l-arginine have been investigated considerably in cancer, trauma (19), and several other infectious diseases, including *Trypanosoma cruzi* (20), *Toxoplasma gondii* (21), *Pseudomonas aeruginosa* (22), *Plasmodium falciparum* (23), *Listeria monocytogenes* (24), and *Mycobacterium tuberculosis* (25) infections, but role of l-arginine in host immune responses against *L. donovani* infection and its biological relevance to disease outcome is obscure. Previous studies reported that trypanosomatids lack a biosynthetic route for l-arginine (26). *Leishmania* parasite cannot synthesize l-arginine *de novo*, indicating that its metabolism depends on extracellular supplies, making l-arginine, an essential amino acid for the growth and survival of the parasite (27, 28). Krassner and Flory reported that l-arginine is an important molecule for the growth of *Leishmania* parasites (29), and these parasites import this amino acid from *in vitro* culture media (29, 30) for their survival. Nonetheless, how the Leishmania parasite utilizes l-arginine inside macrophages and promotes its growth has yet not been clearly elucidated. Polyamine biosynthesis in *Leishmania* parasites takes a convoluted pathway, beginning with the l-arginine scavenged from the host, then translocated to glycosomes by an as yet unexplored permeation process (26). Furthermore, it has also been documented that *in vitro* cultured *Leishmania* parasites can directly attain and employ l-arginine from the extracellular milieu for polyamine production (26, 31). Previously, Castilho-Martins et al. reported that in *L. (L.) amazonensis*, arginine uptake is controlled by transporter-coding mRNA levels and they suggested a mechanism that senses internal arginine concentrations and regulates uptake of l-arginine by augmenting expression of arginine transporter (32). Later, Goldman-Pinkovich et al. reported that parasites respond to the inadequacy of l-arginine by elevating expression and activity of the *Leishmania* arginine transporter (LdAAP3) in addition to numerous other transporters and they proposed that the arginine deprivation response is mediated through a mitogen-activated protein kinase-2-dependent signaling cascade (33). However, the involvement of host pathways by which *Leishmania* can acquire the l-arginine pool within the MΦs remain obscure. Boitz et al. recently reported that arginase is essential for polyamine biosynthesis *de novo* and for promastigote growth in unsupplemented media but not for intracellular amastigotes suggesting that *L. donovani* amastigotes in the parasitophorous vacuole scavenge ornithine and spermidine for their survival (34).

RETRACTED

Several mammalian l-arginine transport systems, encompassing systems y+, Bo+, bo+, and y + L, have been reported (35). The basal level of l-arginine is retained mainly through the y + L system in non-activated MΦs, while transport through the y+ system exacerbates considerably in activated MΦs (36). The cationic amino acid transporter family (CAT) belongs to the y+ system transporter family that comprises four members, CAT-1 to CAT-4, encoded by the *Slc7A1* to *-4* genes, respectively (35). Arginine is transported by the first three members (CAT-1, -2, and -3) of the CAT family (37). CAT-1 is ubiquitously expressed excluding in liver while CAT-3 is rendered only in brain. CAT-2 exists in two isoforms, with CAT-2A being basically expressed in the liver and muscle cells (38) and CAT-2B in the macrophages (39). CAT-2B is induced by cytokines in several cell types, including MΦs and plays a critical role in the modulation of iNOS and arginase activities (40). However, there is limited knowledge on how this transporter directly determines the outcome of *Leishmania* infection. It is reported that in MΦs with impairing l-arginine transporter, NO and polyamine synthesis were diminished upon activation with Th1 and Th2 cytokines, respectively (36), demonstrating that l-arginine accessibility is the impediment control step for both iNOS and arginase.

In the present study, we deciphered the involvement of CAT for the transport of l-arginine in *Leishmania*-infected macrophages and tried to understand the pathways by which l-arginine is utilized. Our study indicated that intra-macrophage survival of *L. donovani* depends on the availability and transport of extracellular l-arginine because intra-macrophage parasite burden was reduced upon inhibition of l-arginine availability and transport either by pharmacological inhibitor or by siRNA-mediated downregulation of the transporter. Furthermore, CAT-2 was observed to be the major isoform associated with l-arginine transport in *L. donovani*-infected macrophages. l-arginine supply regulated the host arginase in *Leishmania* infection. Simultaneously, inhibition of l-arginine transport as well as arginase leads to decreased polyamine production, resulting in decreased parasite survival inside macrophages. Therefore, we hope that understanding the biological role played by arginine deficiency in case of *Leishmania* infection will lead to its early identification and to the design of new and novel treatments.

RETRACTED

## Materials and Methods

### Ethics Statement

All studies were approved by the Institutional Human Ethical Committee of the Rajendra Memorial Research Institute of Medical Sciences (Patna, India). Human monocyte-derived macrophages (hMDM) were isolated from healthy adult individuals after written, informed consent. Routine experimentation with animals was approved by the Institutional Animal Ethical Committee of the Rajendra Memorial Research Institute of Medical Sciences, Patna, India.

### Reagents

THP-1 cell line was purchased from NCCS, Pune, India. Phorbol 12-myristate 13-acetate (PMA), l-arginine, *N*-Ethylmaleimide (NEM; inhibitor of l-arginine transport), L-N^6^-(1-Iminoethyl) lysine dihydrochloride (L-NIL; inhibitor of iNOS), sulfanilamide (component of Griess reagent), and *N*-(1-Naphthyl) ethylenediamine dihydrochloride (NED; component of Griess reagent) were purchased from Sigma-Aldrich (St. Louis, MO, USA). (S)-(2-Boronoethyl)-l-cysteine, HCl (BEC; inhibitor of arginase), and Dansyl chloride were purchase from EMD Millipore, USA. Fetal bovine serum (FBS), OptiMEM, dialyzed FBS, and Lipofectamine RNAiMax reagent were purchased from Invitrogen, USA. siRNAs for CAT-1 (sc-44923), CAT-2 (sc-77441), Arg-1 (sc-29728), Arg-2 (sc-29729), and iNOS (sc-29417) were purchased from Santa Cruz Biotechnology, USA. PCR primers were designed from Avantor, IDT, USA. HRP-conjugated secondary antibodies were purchased from Jackson Laboratory, USA. [^3^H] l-arginine was purchased from PerkinElmer, Singapore. Amersham™ ECL™ Prime Western Blotting Detection Reagent was purchased from GE Healthcare, UK.

### Culture of Parasite

*Leishmania donovani* strain AG83 (MHOM/IN/1983/AG83), used in this study was maintained routinely in golden hamsters by repeated passage to sustain its virulence. Amastigotes were isolated from the spleen of infected hamster and were made to undergo transformation from amastigotes to promastigotes routinely, prior to infection as described earlier (41). *Leishmania* parasites were grown at 22°C in normal RPMI media (Invitrogen, USA) and supplemented with 10% heat-inactivated dialyzed FBS (Invitrogen, USA), 25 mM HEPES, pH 7.4, 4 mM NaHCO_3_, 100 U/ml of penicillin G-sodium (Sigma-Aldrich), and 100 mg/ml of streptomycin (Sigma-Aldrich), and these parasites were used for our experimental purpose. Levels of LPS in parasite stock preparations were found to be below the limit of detection [<0.1 endotoxin U/ml (LAL-test; BioWhittaker, Inc., Walkersville, MD, USA)].

RETRACTED

### Cell Culture and Infection

THP-1 cells, an acute monocytic leukemia-derived human cell line, were maintained in RPMI-1640 (Invitrogen, USA) medium supplemented with 10% heat-inactivated FBS (Invitrogen, USA) and penicillin (100 U/ml), streptomycin (100 mg/ml), and gentamycin (20 µg/ml) at 37°C in humidified air containing 5% CO_2_. The cells were treated with 20 nM phorbol 12-myristate 7-acetate (PMA) for 48 h so as to become matured macrophage-like phenotype and adhered with plastic. Non-adherent cells were removed by washing with RPMI without FBS. The cells were then further incubated in complete RPMI media containing no PMA for 24 h before using it for the experimental purpose.

Blood was collected from healthy donors in heparinized tubes and was processed within 10 min after blood collection. Mononuclear cells were isolated from peripheral blood by density gradient centrifugation over Ficoll-Paque Plus (GE Healthcare, Piscataway, NJ, USA) according to the manufacturer’s instructions. The viability of the mononuclear cells was checked by trypan blue dye exclusion method (~95%). hMDMs were isolated by the method as described previously (42). Briefly, isolated monocytes were cultured overnight in 6-well plates at a density of 2 × 10^6^ cells per well in the presence of macrophage colony-stimulating factor (M-CSF) (300 ng/ml) in RPMI medium with 10% FBS. Non-adherent cells were repeatedly washed, and cells were allowed to differentiate into MDMs in the presence of M-CSF and 10% FBS. Differentiated MDMs were harvested after 96 h.

The THP-1 or hMDMs were infected with *Leishmania* parasites for 6 hs at macrophage/parasite multiplicities of 1:10. The unbound parasites were removed by washing with RPMI without FBS followed by additional incubation of up to 48 h in complete RPMI medium. The cells were then fixed followed by staining with May-Grunwald Giemsa and observation under bright field microscope at 100× with oil immersion. Parasite load was determined by counting the number of amastigotes per 100 macrophages and percent infectivity was calculated by counting the number of infected cells (43). The results were expressed as mean ± SD of three independent experiments performed in triplicate.

### Transfection

THP-1 cells (1 × 10^6^) or hMDMs were seeded in 6-well plate. Fresh siRNA transfection reagent containing siRNA (final concentration 25 nM), optiMEM, and lipofectamine RNAiMax was prepared by the protocol as described previously (44). The above reagent (200 µl) was added to each well and cultured for 6 h. Then, the supernatant was aspirated and cells were further cultured with fresh complete growth medium for 12–15 h before any inhibitor treatment. Confirmation of siRNA-mediated downregulation of target gene was evaluated by western blot analysis. Control cells were without siRNA.

RETRACTED

### Measurement of Arginase Activity

Arginase activity in THP-1 or hMDM lysates were measured using a micromethod as described previously (45, 46). Briefly, after incubations, cells were lysed with 0.1% Triton X-100. After 30 min on a shaker, 25 mM Tris–HCl were added to the lysate. Then, to this lysate, 10 mM MnCl_2_ were added, and the enzyme was activated by heating for 10 min at 56°C. Arginine hydrolysis was supervised by incubating the lysate with 0.5 M l-arginine (pH 9.7) for 15–20 min at 37°C. The reaction was stopped with H_2_SO_4_ (96%)/H_3_PO_4_ (85%)/H_2_O (1/3/7, v/v/v) followed by addition of α-isonitrosopropiophenone (dissolved in 100% ethanol) and heating at 95°C for 30 min. The concentration of urea produced was quantified at 540 nm. Protein concentration was measured by BCA method [Pierce Thermo Fisher Scientific]. One unit of enzyme activity was defined as the amount of enzyme that catalyzes the formation of 1 µmol urea/min. BEC (200 µM) was used as an inhibitor of arginase as described previously (43, 47). Each measurement was performed in triplicate and the data were expressed as mean ± SD of three independent experiments.

### Measurement of NO

Nitrite $\left({\text{NO}}_{\text{2}}^{-}\right)$ accumulation was used as an indicator of NO production and measured by using the Griess reagent (48). THP-1 or hMDM culture supernatants were collected after 48 h of incubation. Equal volume of supernatants and Griess reagent [1% sulphanilamide/0.1% *n*-(1-napthyl) ethylenediamine dihydrochloride/2.5% H_3_PO_4_] were mixed and incubated for 10 min at room temperature. Absorbance was recorded at 540 nm in a plate reader (Thermo Multiscan, USA). Nitrite concentration was estimated using NaNO_2_ as standard. L-NIL (100 ng/ml) was used as an inhibitor of iNOS as described previously (49).

### Semi-Quantitative RT-PCR and Quantitive Real-time PCR

RNA was extracted from macrophages (THP-1 and hMDM), and c-DNA was prepared from 20 µg of total RNA using c-DNA synthesis kit (Invitrogen). The c-DNAs were used in PCR amplification of l-arginine transporters, such as CAT-1, CAT-2A, CAT-2B, arginine metabolizing enzymes such as Arg-1, Arg-2, iNOS, and cytokines such as IL-10, IL-12 and TNF-α using gene-specific primers. After initial denaturation at 94°C for 5 min, targeted genes were amplified (94°C for 45 s, 56°C or 58°C for 30 s, and 72°C for 1 min) for 25 amplification cycles followed by a final extension at 72°C for 10 min. The PCR products were run on ethidium bromide stained 1.5% agarose gel and finally documented and quantified in gel documentation system (Bio-Rad) associated Quantity One software. All the PCR products were normalized with respect to GAPDH transcript and expressed as fold change. Each measurement was performed in triplicate and one of the representative gel image was shown. The data were expressed as mean ± SD of three independent experiments.

RETRACTED

These semi-quantitative data were further validated by quantitative real-time PCR, which was performed in the LightCycler 480 (Roche) using SYBR green (Roche) chemistry as described previously (50). The cycling conditions were as follows: 1 cycle at 95°C for 3 min and 40 cycles of 95°C for 15 s (denaturation), 58°C for 30 s (annealing), and 72°C for 30 s (extension). The fluorescence signal was captured at the end of each cycle using the SYBR channel (490 nm wavelength for excitation and 525 nm wavelength for emission). Results were analyzed by LightCyclerR 480 relative quantification software (Roche) and expressed as the target/reference ratios of each sample, normalized by the target/reference ratio of the calibrator. Here, the target/reference value of uninfected macrophages was used as calibrator and GAPDH was used as reference. The primers used for both semi-quantitative RT-PCR and quantitative real-time PCR are summarized in Table S1 in Supplementary Material.

### Western Blotting

After individual incubations were over, protein was isolated from MΦs (THP-1 and hMDM). 50 µg of each protein were separated by electrophoresis on 12% SDS-polyacrylamide gel and transferred onto PVDF membrane (43). Membrane was washed with 1× TBST solution thrice and blocked with 3% BSA for 2 h at room temperature. Blocked membrane was washed in TBST solution thrice and then was incubated with monoclonal primary antibody against CAT-1, CAT-2, Arg-1, Arg-2, and iNOS. Horseradish peroxidase-conjugated secondary antibody was used, and the protein band was visualized by enhanced chemiluminescence reaction, normalized with respect to GAPDH and expressed as fold change. Each measurement was performed in triplicate and one of the representative gel image was shown. The data were expressed as mean ± SD of three independent experiments.

### Measurement of Polyamines

Poyamines (putrescine and spermidine) were identified and quantified by a prederivatization method using high performance liquid chromatography (HPLC) as described by Balaña-Fouce et al. (51). Briefly, after incubations, both uninfected and infected macrophages were harvested, washed twice with PBS (pH 7.4), and the last pellet was disintegrated with 5% trichloroacetic acid (w/v) overnight. The extracts were centrifuged (10,000 *g*, 15 min), and the supernatant was neutralized with a saturated NaHCO_3_ solution. The mixture was incubated with a solution containing 20 mg dansyl chloride/ml (Merck) in acetone (Merck. HPLC grade) at 50°C for overnight. The dansylated polyamines were extracted twice with toluene (Merck, HPLC grade), evaporated under nitrogen stream and the precipitate was dissolved in 1 ml of acetonitrile (Merck, HPLC grade), before analysis by HPLC on a C^18^ reverse-phase column (Shimadzu, Japan). Dansylated polyamines were quantified with a spectrofluorimeter at excitation of 330 nm and emission at 510 nm. The peak areas, retention times were recorded and calculated by a PC Integration Pack Programme. The level of polyamines were expressed as nmol per 10^6^ cells. There were three replicates in each test, and the data were the mean ± SD of three independent observations.

RETRACTED

### Measurement of l-Arginine Transport

Uptake of l-arginine in macrophages were measured using the protocol described elsewhere (32) with minor modifications. Briefly, after incubation, THP-1 or hMDM (1 × 10^6^ macrophages/ml) were pelleted down and washed with cold Earle’s Balanced Salt Solution (EBSS) containing 137 mM NaCl, 26 mM NaHCO_3_, 5 mM KCl, 1.8 mM CaCl_2_, 1 mM NaH_2_PO_4_, 0.8 mM MgSO_4_, and 5.5 mM glucose twice followed by resuspension in [^3^H]-l-arginine (5 μCi/ml) using stock from 1 mCi/ml (specific activity-51.5 Ci/mmole) (PerkinElmer, Singapore) at 25°C. Uptake was stopped after 8 min by adding 50 mM of ice-cold l-arginine (non-radioactive). Macrophages were then washed twice with EBSS, lysed in lysing solution (0.1% SDS, 100 mM NaOH). The incorporated radioactivity inside cell was estimated using liquid scintillation counter (Tri-Carb 2810 TR, PerkinElmer, USA). Uptake was expressed as nmol/10^6^ cells/min. NEM (CAT specific inhibitor, 250 µM) was used as an inhibitor of l-arginine transport as described previously (52, 53). Each measurement was performed in triplicate and data were expressed as mean ± SD of three independent experiments.

### ELISA

The level of cytokines IL-10, IL-12, and TNF-α in the supernatant of THP-1 macrophages were determined using commercial BD OptEIA ELISA kits (BD, San Jose, CA, USA) according to manufacturer’s protocol as described previously (41). The BD OptEIA test is a solid phase sandwich enzyme-linked immunosorbent assay (ELISA). Required quantities of strips were taken and 50 µl of ELISA diluent was added to each well. After that, 100 µl of standard/sample was added and incubation at RT was done for 2 h followed by five times washing. 100 µl of detection antibody was then added followed by 1 h incubation. Washing was done seven times, and 100 µl of TMB One-Step Substrate was added. Incubation was done for 30 min at RT and then 50 µl of stop solution was added to stop the reaction and quantitative measurement was done by taking absorbance at 450 nm. Cytokine concentrations were estimated from respective standard curve and expressed as pg/ml.

RETRACTED

### Statistical Analysis

We analyzed our data using Graph Pad Prism (Version 6.0, GraphPad Software, USA). Each experiment was repeated three times in separate sets and the results were expressed as Mean ± SD. Statistical differences were determined using Mann–Whitney *U* test for comparing two groups or Kruskal–Wallis with Dunn’s multiple comparison test for comparing three or more groups. *p* ≤ 0.05 were considered significant.

## Results

### l-Arginine Availability Regulates *Leishmania* Viability inside Macrophages

In our previous study, we have shown that l-arginine is an important amino acid for the survival of *Leishmania* promastigotes. In that study, we observed that the viability and the cell proliferation were greatly diminished when parasites were grown in l-arginine-depleted media (43). In the present study, the same phenomena were examined in *Leishmania* parasites inside macrophages. Macrophages (THP-1 and hMDM) were cultured in l-arginine-depleted and l-arginine-supplemented RMPI medium separately and then infected with *L. donovani* parasite. However, macrophages were never switched from l-arginine-replete to l-arginine-depleted conditions. It was observed that macrophage viability was not altered upon l-argininie deprivation (data not shown). Further, it was observed that both parasite load (Figures 1A,B,D) and percent infectivity (Figures 1A,C,E) was increased at 48 h when compared to 6 and 24 h. Simultaneously, both parasite load and percent infectivity was significantly higher in l-arginine-supplemented media compared to l-arginine-depleted media at 24 and 48 h (*p* ≤ 0.05). However, no significant change in parasite load or percent infectivity were observed at 6 h time point upon l-arginine deprivation from the culture media. Parasite load was found to be significantly reduced (~2.04-fold at 24 h and ~2.27-fold at 48 h; *p* ≤ 0.05) in case of THP-1 macrophages grown in l-arginine-depleted medium compared to l-arginine-supplemented medium (Figures 1A,B). Similarly, significant decrease in parasite load was also observed (~2.16-fold at 24 h and ~2.29-fold at 48 h; *p* ≤ 0.05) when hMDM were cultured in l-arginine-depleted medium compared to l-arginine-supplemented medium (Figure 1D). On the other hand, percent infectivity was significantly reduced (~1.5-fold at 24 h and ~1.6-fold at 48 h *p* ≤ 0.05) when THP-1 macrophages were grown in l-arginine-depleted medium compared to l-arginine-supplemented medium (Figures 1A,C). Simultaneously, in case hMDM, percent infectivity was found to be reduced by ~1.65-fold at 24 h and ~1.6-fold at 48 h when macrophages were cultured in l-arginine-depleted medium compared to l-arginine-supplemented medium (Figure 1E). Therefore, these findings suggested that the availability of l-arginine in the culture media promotes parasite survival inside macrophages. However, in its absence, parasite growth was significantly reduced indicating that l-arginine is an important amino acid for the survival of *Leishmania* inside macrophages.

RETRACTED

**Figure 1:** Effect of l-arginine availability on survival of *Leishmania* parasite inside macrophages. THP-1 monocyte-derived MΦs **(A,B,C)** and human monocyte-derived macrophages (hMDM) **(D,E)** (5 × 10^4^ cells/ml) were grown in l-arginine-supplemented and l-arginine-depleted RPMI medium followed by infection with *Leishmania donovani* (multiplicity of infection 1:10) for 6, 24, and 48 h. Intracellular parasites were visualized by staining the cells with Giemsa followed by optical microscopy at 100× oil immersion **(A)**. The horizontal bar indicates 5 µm size. The parasite load was measured by counting the number of intracellular amastigotes per 100 macrophages **(B,D)**. The rate of infection was analyzed by counting the percent infected macrophages **(C,E)**. Each experiment was repeated three times. Each determination was made in triplicate and the values were expressed as mean ± SD for three independent experiments. Mann–Whitney *U* test was used to evaluate statistical significance for comparing two groups; *p < 0.05; **p < 0.005.

### *Leishmania* Infection Upregulates l-Arginine Transport through CAT-2 Transporter

In the present study, we wanted to observe the effect of l-arginine starvation from extracellular milieu on the expression of macrophage l-arginine transporters (CAT-1, CAT-2) in normal and infected condition. We also measured the amount of l-arginine transport during *Leishmania* infection in presence or absence of l-arginine in the culture medium. THP-1-derived macrophages and hMDM were cultured in l-arginine-depleted as well as l-arginine-supplemented RPMI media and infected with *L. donovani* parasite for 48 h. The expression of CAT-1 and CAT-2 (CAT-2A and CAT-2B) were checked at the transcript level by semi-quantitive RT-PCR as well as quantitive real-time PCR and translational level by western blot. No significant change in CAT-1 or CAT-2A expression was observed in case of *Leishmania* infection either in l-arginine-depleted or l-arginine-supplemented condition (Figures 2A–E).

RETRACTED

**Figure 2:** Effect of *Leishmania* infection on expression of CAT-1 and CAT-2. THP-1 monocyte-derived MΦs **(A,B,D)** and human monocyte-derived macrophages (hMDM) **(C,E)** (1 × 10^6^ cells/ml) were grown in l-arginine-supplemented and l-arginine-depleted RPMI medium followed by infection with *Leishmania donovani* (multiplicity of infection 1:10) for 48 h. The expression of CAT-1 and CAT-2 (CAT-2A and CAT-2B) were evaluated at the transcript level by semi-quantitative RT-PCR **(A)** and real-time PCR **(B,C)** and protein level by western blotting **(D,E)**. The intensity of the bands were quantified by densitometry in Quantity one software. Each experiment was repeated three times. Semi-QRT PCR gel images and western blots are representative of three experiments. Densitometric plots are shown adjacent to the gel images. Data are mean ± SD (*n* = 3) (*p < 0.05; **p < 0.001; ns, non-significant) (Mann–Whitney *U* test).

However, from the semi-quantitive PCR data, it was observed that in case of *Leishmania* infection to THP-1, the expression of CAT-2B transcript was increased by ~2.8-fold in l-arginine-supplemented condition and ~5.8-fold in l-arginine-depleted condition (Figure 2A). Similar results were observed when we checked the expression of CAT-2B by quantitive real-time PCR. In this case, the expression of CAT-2B transcript was increased by ~2.7-fold in l-arginine-supplemented condition and ~6.7-fold in l-arginine-depleted condition (Figure 2B). Comparative analysis indicated that CAT-2B transcript is significantly increased upon l-arginine deprivation (~2.1-fold, *p* ≤ 0.005 in case of semi-QRT PCR and ~2.5-fold, *p* ≤ 0.005 in case of quantitive real-time PCR) in case of *Leishmania* infection (Figures 2A,B). The expression of CAT-2B in *Leishmania*-infected hMDM was further checked by real-time PCR. It was observed that in case of *Leishmania* infection, the expression of CAT-2B transcript was increased by ~2.5-fold in l-arginine-supplemented condition and ~5.8-fold in l-arginine-depleted condition (Figure 2C). Comparative analysis indicated that l-arginine deprivation led to significant increase (~2.3-fold, *p* ≤ 0.005) in CAT-2B transcript in *Leishmania*-infected macrophages compared to l-arginine supplementation (Figure 2C). Simultaneously, from the western blot data, it was also observed that deprivation of l-arginine led to significant increase (~2.8-fold, *p* ≤ 0.005) in CAT-2 in *Leishmania*-infected macrophages when compared to l-arginine supplementation (Figure 2D).

RETRACTED

The expression of CAT-2 in *Leishmania*-infected hMDM were also checked by western blot and comparative analysis indicated that CAT-2 is significantly increased in case of *Leishmania* infection upon l-arginine deprivation (~2.1-fold, *p* ≤ 0.005) compared to l-arginine supplementation (Figure 2E).

The expression of CAT-1 and CAT-2 was further assessed in *Leishmania*-infected macrophages pretreated with inhibitor of l-arginine transport (NEM) both at the transcript and translational level. Surprisingly, no significant change in CAT-1 or CAT-2 expression was observed in case of NEM pretreatment either at the transcript or protein level (Figures 3A–E).

**Figure 3:** Effect of NEM on expression of CAT-1 and CAT-2 in *Leishmania donovani*-infected macrophages. THP-1 MΦs **(A,B,D)** and human monocyte-derived macrophages (hMDM) **(C,E)** were left untreated or preincubated with NEM (250 µM) for 10 min followed by infection with *L. donovani* for 48 h. The expression of CAT-1 and CAT-2 (CAT-2A and CAT-2B) were evaluated at the transcript level by semi-quantitative RT-PCR **(A)** and real-time PCR **(B,C)** and protein level by western blotting **(D,E)**. The intensity of the bands were quantified by densitometry in Quantity one software. Each experiment was repeated three times. Semi-QRT PCR gel images and western blots are representative of three experiments. Densitometric plots are shown adjacent to the gel images. Data are mean ± SD (*n* = 3) (*p < 0.05; **p < 0.001; ns, non-significant) (Mann–Whitney *U* test).

Uptake of l-arginine in uninfected and infected THP-1 and hMDM were measured by radioactivity incorporation. It was observed that in case of *Leishmania* infection to THP-1, l-arginine transport was increased by ~2.7-fold in normal condition and ~4.2-fold in case of l-arginine deprivation (Figure 4A). However, at the same time, comparative analysis indicated that l-arginine deprivation leads to significant increase (~2.3-fold, *p* ≤ 0.005) in l-arginine transport in *Leishmania-*infected THP-1 (Figure 4A).

**Figure 4:** Effect of *Leishmania* infection on l-arginine transport. THP-1 monocyte-derived MΦs **(A)** and human monocyte-derived macrophages (hMDM) **(B)** (1 × 10^6^ cells/ml) were grown in l-arginine-supplemented and l-arginine-depleted RPMI medium followed by infection with *Leishmania donovani* (multiplicity of infection 1:10) for 48 h. In another experiment, THP-1 MΦs **(C)** and hMDM **(D)** were left untreated or preincubated with NEM (250 µM) for 10 min followed by infection with *L. donovani* for 48 h. In a separate experiment, THP-1 MΦs **(E)** and hMDM **(F)** (1 × 10^6^ cells/ml) were transfected with control siRNA, CAT-1 or CAT-2 siRNA followed by infection with *L. donovani* for 48 h. Arginine transport was measured after incubating the cells with 1 μCi/ml of [^3^H] l-arginine uptake solution for 8 min followed by counting the incorporation of [^3^H] l-arginine in liquid scintillation counter **(A–F)**. Each experiment was repeated three times. Each determination was made in triplicate and the values were expressed as mean ± SD for three independent experiments. Kruskal–Wallis with Dunn’s multiple comparison test was used to evaluate statistical significance for comparing three or more groups; *p < 0.05; **p < 0.005; ns, non-significant.

RETRACTED

Simultaneously, when we measured l-arginine transport in *Leishmania*-infected hMDM, it was observed that in case of *Leishmania* infection, l-arginine transport was increased by ~2.3-fold in normal condition and ~3.6-fold in case of l-arginine deprivation condition (Figure 4B). Furthermore, comparative analysis indicated that l-arginine transport is significantly increased in case of *Leishmania* infection upon l-arginine deprivation (~1.8-fold, *p* ≤ 0.005) compared to l-arginine-supplemented condition (Figure 4B).

The effect of NEM on macrophage l-arginine transport was further checked. It was observed that NEM pretreatment decreased l-arginine transport by ~2.4-fold in *Leishmania*-infected THP-1 macrophages (Figure 4C) and ~2.0-fold in *Leishmania*-infected hMDM (Figure 4D).

Further, to confirm that CATs are the main transporters for l-arginine in macrophages, we downregulated macrophage CAT-1 and CAT-2 by siRNA-mediated transfection and then infected with *Leishmania* parasite. It was observed that silencing of CAT-1 or CAT-2 had no significant effect on l-arginine transport in uninfected macrophages (Figures 4E,F). Simultaneously, CAT-1 knock down showed no significant decrease in l-arginine transport in *Leishmania*-infected THP-1 macrophages or hMDM. On the other hand, CAT-2 silencing leads to significant decrease (~2.6-fold; *p* ≤ 0.005) in l-arginine transport in *Leishmania*-infected macrophages compared to normal infected macrophage (Figures 4E,F). Hence, our results suggested that CAT-2 is the main isoform associated with l-arginine transport in *Leishmania*-infected macrophages. Our study pointed out that as *Leishmania* is auxotroph for l-arginine, it modulates the host to upregulate the expression of CAT, thereby increases l-arginine uptake and utilizes this amino acid for their survival inside macrophages.

### Inhibition of Macrophage l-Arginine Transport Limits *Leishmania* Survival inside Macrophages

Further, we studied the effect of inhibition of l-arginine transport upon survival of *Leishmania* parasite inside macrophages. For this, we pretreated both THP-1 macrophages and hMDM with NEM (250 µM) and infected with *Leishmania* parasite for 48 h and measured the parasite load and percent infectivity. A ~2.4-fold reduction in parasite load (Figures 5A,B) and ~2.3-fold reduction in percent infectivity (Figures 5A,C) was observed when THP-1 macrophages were pretreated with NEM. Similar results were observed with the use of hMDM. In this case ~2.8-fold reduction in parasite load (Figure 5B) and ~2.7-fold reduction in percent infectivity (Figure 5C) was observed when hMDM were pretreated with NEM.

RETRACTED

**Figure 5:** Effect of inhibition of macrophage l-arginine transport on survival of *Leishmania* inside MΦ. THP-1 monocyte-derived MΦs **(A–C)** and human monocyte-derived macrophages (hMDM) **(B,C)** (5 × 10^4^ cells/ml) were either left untreated or preincubated with 250 µM NEM for 10 min followed by infection with *Leishmania donovani* (multiplicity of infection 1:10) for 48 h. In a separate experiment, THP-1 MΦs **(D,E,F)** and hMDM **(E,F)** (1 × 10^6^ cells/ml) were transfected with control siRNA, CAT-1 or CAT-2 siRNA followed by infection with *L. donovani* for 48 h. Intracellular parasites were visualized by staining the cells with Giemsa followed by optical microscopy at 100× oil immersion **(A,D)**. The horizontal bar indicates 5 µm size. The parasite load was measured by counting the number of intracellular amastigotes per 100 macrophages **(B,E)**. The rate of infection was analyzed by counting the percent infected macrophages **(C,F)**. Each experiment was repeated three times. Each determination was made in triplicate and the values were expressed as mean ± SD for three independent experiments. Mann–Whitney *U* test was used to evaluate statistical significance for comparing two groups. Kruskal–Wallis with Dunn’s multiple comparison test was used to evaluate statistical significance for comparing three or more groups; *p < 0.05; **p < 0.005; ns, non-significant.

Parasite load and percent infectivity were further measured in CAT-1 and CAT-2 siRNA transfected *Leishmania*-infected THP-1 macrophages and hMDM. It was observed that silencing of CAT-1 had no significant effect on parasite load and percent infectivity. However, CAT-2 knock down decreased the parasite load by ~4.7-fold (Figures 5D,E) and percent infectivity by ~2.4-fold (Figures 5D,F) in *Leishmania*-infected THP-1 macrophages compared to control siRNA transfected macrophages. Significant reduction in parasite load and percent infectivity were also observed in case of hMDM CAT-2 knock down (Figures 5E,F). Therefore, our study indicated that l-arginine transport is critically involved in the regulation of parasite survival inside macrophages.

RETRACTED

### l-Arginine Availability Regulates Expression of Arginase and iNOS in Infected Macrophages

The effect of l-arginine availability in regulation of arginase–iNOS balance in *Leishmania*-infected macrophages was investigated. We cultured THP-1 macrophages and hMDM in l-arginine-depleted as well as l-arginine-supplemented RPMI media, infected with *L. donovani* parasite for 48 h and checked the expression of Arg-1, Arg-2, and iNOS at the transcript level by semi-quantitive RT-PCR and quantitive real-time PCR. The expression of macrophage Arg-1 and Arg-2 was increased by ~2.3-fold and ~1.8–fold, respectively, upon *Leishmania* infection in case of normal (l-arginine supplementation) condition (Figure 6A). However, in case of l-arginine deprivation, no significant increase in Arg-1 or Arg-2 expression was observed upon *Leishmania* infection (Figure 6A). Comparative analysis indicated significant decrease in Arg-1 (~2.7-fold; *p* ≤ 0.005) and Arg-2 (~1.8-fold; *p* ≤ 0.05) expression in infected macrophages upon l-arginine deprivation (Figure 6A). However, no significant change in iNOS expression was observed upon l-arginine deprivation in case of *Leishmania* infection. Similar results were observed when the expression of these genes was studied by real-time PCR (Figure 6B).

**Figure 6:** Effect of inhibition of l-arginine availability on Arg-1, Arg-2, and inducible nitric oxide synthase (iNOS) expression in case of *Leishmania* infection. THP-1 monocyte-derived MΦs (1 × 10^6^ cells/ml) were grown in l-arginine-supplemented and l-arginine-depleted RPMI medium followed by infection with *Leishmania donovani* (multiplicity of infection 1:10) for 48 h **(A,B)**. In another experiment, THP-1 monocyte-derived MΦs (1 × 10^6^ cells/ml) were left untreated or preincubated with NEM (250 µM) for 10 min followed by infection with *L. donovani* for 48 h **(C,D)**. In a separate experiment, THP-1 monocyte-derived MΦs (1 × 10^6^ cells/ml) were transfected with control siRNA, CAT-1, or CAT-2 siRNA followed by infection with *L. donovani* for 48 h **(E,F)**. The expression of Arg-1, Arg-2, and iNOS were determined at the transcript level by semi-quantitative RT-PCR **(A,C,E)** and real-time PCR **(B,D,F)**. The intensity of the bands was quantified by densitometry using Quantity one software. Each experiment was repeated three times. Each determination was made in triplicate and the values were expressed as mean ± SD for three independent experiments. Semi-QRT PCR gel images are representative of three experiments. Densitometric plots are shown below the gel images. Kruskal–Wallis with Dunn’s multiple comparison test was used to evaluate statistical significance for comparing three or more groups; *p < 0.05; **p < 0.005; ns, non-significant.

RETRACTED

The expression of these genes were further checked by limiting l-arginine availability through blockade of l-arginine transporter (CATs) by NEM (CAT specific inhibitor) and siRNA-mediated downregulation. NEM pretreatment decreased the expression of Arg-1 by ~2.0-fold and Arg-2 by ~1.5-fold in infected macrophages (Figure 6C). Similar results were observed when the expression of these genes were studied by real-time PCR (Figure 6D).

Furthermore, silencing of CAT-1 decreased the expression of Arg-1 by ~1.96-fold and had no significant effect on expression of Arg-2 and iNOS in *Leishmania*-infected macrophages. However, CAT-2 knock down decreased Arg-1 expression by ~2.3-fold, Arg-2 expression by ~1.9–fold, and iNOS expression by ~2.0-fold in *Leishmania*-infected macrophages compared to control siRNA transfected macrophages (Figure 6E). Simultaneously, when we checked the expression of these genes by real-time PCR, we also observed that silencing of CAT-1 decreased Arg-1 expression by ~2.0-fold whereas it had no significant effect on Arg-2 and iNOS expression in *Leishmania*-infected macrophages. On the other hand, CAT-2 knock down decreased the expression of Arg-1 by ~2.7-fold and Arg-2 by ~1.9-fold in *Leishmania*-infected macrophages (Figure 6F). Therefore, our results indicated that l-arginine availability and transport is critically involved in the regulation of Arg-1, Arg-2, and iNOS expression in *Leishmania*-infected macrophages.

The reciprocal regulation of arginase and iNOS in case of *Leishmania* infection was further evaluated at the transcript and translational level using an inhibitor of arginase (BEC) and iNOS (L-NIL). From the semi-quantitive RT-PCR data, it was observed that inhibition of iNOS increased Arg-1 transcript by ~1.9-fold and Arg-2 by ~1.9-fold, whereas, arginase inhibition upregulated iNOS transcript by ~4.6-fold in infected macrophages (Figure 7A). Simultaneously, real-time PCR data further confirmed that inhibition of iNOS led to significant increase in Arg-1 (~1.7-fold; *p* ≤ 0.05) and Arg-2 (~1.7-fold; *p* ≤ 0.05) transcript, whereas, arginase inhibition led to increased iNOS (~4.6-fold; *p* ≤ 0.05) transcript in *Leishmania*-infected macrophages (Figure 7B).

**Figure 7:** Regulation of Arg-1, Arg-2, and inducible nitric oxide synthase (iNOS) expression in case of *Leishmania donovani* infection. THP-1 monocyte-derived MΦs (1 × 10^6^ cells/ml) were either left untreated or preincubated with BEC (200 µM) or L-NIL (100 ng/ml) for 3 h followed by infection with *L. donovani* for 48 h **(A–C)**. The expression of Arg-1, Arg-2, and iNOS was determined at the transcript level by semi-quantitative RT-PCR **(A)** and real-time PCR **(B)** and protein level by western blotting **(C)**. The intensity of the bands was quantified by densitometry using Quantity one software. Each experiment was repeated three times. Each determination was made in triplicate and the values were expressed as mean ± SD for three independent experiments. Semi-QRT PCR gel images and western blots are representative of three experiments. Densitometric plots are shown adjacent to the gel images. Kruskal–Wallis with Dunn’s multiple comparison test was used to evaluate statistical significance for comparing three or more groups; *p < 0.05; **p < 0.005.

RETRACTED

In accordance with the semiQ-RT PCR and real-time PCR result, when we measured the protein level by western blot, we observed that the expression of Arg-1 was increased by ~2.5-fold and Arg-2 by ~2.1-fold upon *Leishmania* infection (Figure 7C). Arginase inhibition increased the iNOS expression by ~2.1-fold, whereas, inhibition of iNOS increased Arg-1 expression by ~1.6-fold and Arg-2 by ~1.8-fold in *Leishmania*-infected macrophages compared to normal infected macrophages (Figure 7C). Therefore, our study indicated that both Arg-1 and Arg-2 are upregulated at the transcript and translational level in case of *Leishmania* infection and Arg-1 is the major isoform associated with *L. donovani* infection. As downregulation of Arg-1 and Arg-2 increased the iNOS level, it is obvious that Arg-1/Arg-2-iNOS balance play a crucial role in regulation of each other and thereby determining the outcome of *Leishmania* infection.

Arginase activity at the enzymatic level was further measured in case of *Leishmania* infection upon l-arginine deprivation. Arginase activity was found to be increased by ~2.7- and ~1.6-fold in *Leishmania*-infected THP-1 macrophages compared to uninfected macrophages in case of l-arginine supplementation condition and l-arginine depletion condition, respectively (Figure 8A). Further, comparative analysis indicated significant decrease in arginase activity (~2.7-fold; *p* ≤ 0.005) in *Leishmania*-infected THP-1 macrophages upon l-arginine deprivation (Figure 8A). Similar results were observed with hMDM. In this case, significant decrease in arginase activity (~2.1-fold; *p* ≤ 0.005) was also observed in infected macrophages upon l-arginine deprivation (Figure 8A).

**Figure 8:** Effect of inhibition of l-arginine availability on regulation of arginase activity and nitric oxide production in macrophages infected with *Leishmania donovani*. THP-1 monocyte-derived MΦs and human monocyte-derived macrophages (hMDM) (1 × 10^6^ cells/ml) were grown in l-arginine-supplemented and l-arginine-depleted RPMI medium followed by infection with *L. donovani* (multiplicity of infection 1:10) for 48 h **(A,D)**. In a separate experiment, both THP-1 monocyte-derived MΦs and hMDM (1 × 10^6^ cells/ml) were left untreated or preincubated with 250 µM NEM for 10 min followed by infection with *L. donovani* for 48 h **(B,E)**. In another experiment, both THP-1 monocyte-derived MΦs and hMDM (1 × 10^6^ cells/ml) were transfected with control siRNA, CAT-1, or CAT-2 siRNA followed by infection with *L. donovani* for 48 h **(C,F)**. Arginase activity in MΦs was assessed spectrophotometrically by the method as described in Section “Materials and Methods.” The protein content was measured by BCA method, and the enzyme activity was expressed as mU/mg protein **(A–C)**. Extracellular nitrite level was measured by Griess method using NaNO_2_ as standard **(D–F)**. Each experiment was repeated three times. Each determination was made in triplicate and the values were expressed as mean ± SD for three independent experiments. Kruskal–Wallis with Dunn’s multiple comparison test was used to evaluate statistical significance for comparing three or more groups; *p < 0.05; **p < 0.005; ns, non-significant.

RETRACTED

Simultaneously, inhibition of l-arginine transport by NEM decreased arginase activity by ~2.4-fold and ~2.43-fold in infected THP-1macrophages and hMDM, respectively, when compared to untreated infected macrophages (Figure 8B).

Arginase activity was further measured in CAT-1 and CAT-2 knock down *Leishmania*-infected macrophages. Our results indicated that silencing of CAT-1 had no significant effect on arginase activity in both *Leishmania*-infected THP-1 and hMDM (Figure 8C). On the other hand, CAT-2 knock down led to significant decrease in arginase activity (~2.3-fold; *p* ≤ 0.005 in THP-1 and ~2.6-fold; *p* ≤ 0.005 in hMDM) in infected macrophages compared to control siRNA transfected *Leishmania*-infected macrophages (Figure 8C).

However, while measuring the NO level, no significant change in NO level was observed in case of *Leishmania* infection upon l-arginine deprivation (Figure 8D). Pretreatment of NEM also had no significant effect on NO level in *Leishmania*-infected macrophages (Figure 8E). NO level was further measured in CAT-1 and CAT-2 siRNA transfected *Leishmania*-infected macrophages and similar results were observed (Figure 8F). Therefore, our results confirmed that l-arginine availability and transport is critically involved in the regulation of arginase activity without altering NO production in *Leishmania*-infected macrophages.

RETRACTED

### l-Arginine Availability and Transport Regulates Polyamine Production

*Leishmania* parasites and all other members of the trypanosomatid family depend on polyamines for growth and survival. As, l-arginine is the precursor molecule for synthesis of polyamines, trypanothiones, and tryparedoxin, the effect of l-arginine availability and transport on regulation of polyamine production for survival of *Leishmania* parasite inside macrophages was investigated. So, we cultured THP-1 macrophages in both l-arginine-depleted and l-arginine-supplemented RPMI media, infected with *L. donovani* and measured the putrescine and spermidine content. Putrescine level was found to be increased by ~3.0-fold and ~1.5-fold in *Leishmania*-infected macrophages compared to uninfected macrophages grown in l-arginine-supplemented and l-arginine-depleted media, respectively (Figure 9A). At the same time, spermidine level was increased by ~2.1-fold and ~1.6-fold (Figure 9B) upon l-arginine supplementation and l-arginine depletion condition, respectively, in infected macrophages. Simultaneously, when we compared the level of polyamines, we observed that putrescine (Figure 9A) and spermidine levels (Figure 9B) were significantly decreased (~2.8-fold, *p* ≤ 0.05 for putrescine and for spermidine ~1.8-fold; *p* ≤ 0.05) in l-arginine-depleted infected macrophages compared to l-arginine-supplemented macrophages.

**Figure 9:** Effect of inhibition of l-arginine availability on regulation of polyamine production in *Leishmania donovani*-infected macrophages. THP-1 monocyte-derived MΦs (1 × 10^6^ cells/ml) were grown in l-arginine-supplemented and l-arginine-depleted RPMI medium followed by infection with *L. donovani* (multiplicity of infection 1:10) for 48 h **(A,B)**. In a seperate experiment, THP-1 MΦs (1 × 10^6^ cells/ml) were either left untreated or preincubated with 250 µM NEM for 10 min followed by infection with *L. donovani* for 48 h **(C,D)**. In another experiment, THP-1 MΦs (1 × 10^6^ cells/ml) were transfected with control siRNA, CAT-1 or CAT-2 siRNA followed by infection with *L. donovani* for 48 h **(E,F)**. The polyamines (putrescine and spermidine) were extracted by TCA precipitation followed by dansyl chloride derivatization, separation by reverse-phase high performance liquid chromatography as described in “Materials and Methods.” Dansylated putrescine **(A,C,E)** and dansylated spermidine **(B,D,F)** were quantified by fluorescence spectrometry. Each experiment was repeated three times. Each determination was made in triplicate and the values were expressed as mean ± SD for three independent experiments. Kruskal–Wallis with Dunn’s multiple comparison test was used to evaluate statistical significance for comparing three or more groups; *p < 0.05; **p < 0.005; ns, non-significant.

RETRACTED

Polyamine level was further measured in *Leishmania*-infected macrophages pretreated with l-arginine transporter inhibitor. It was observed that NEM pretreatment decreased putrescine level by ~2.8-fold (Figure 9C) and spermidine level by ~1.9-fold (Figure 9D) in infected macrophages compared to untreated infected macrophages. Putrescine level was found to be increased by ~3.0-fold, ~3.1–fold, and ~1.5-fold (Figure 9E) while spermidine level by ~2.2-fold, ~2.0–fold, and ~1.6-fold (Figure 9F) in control siRNA transfected, CAT-1 siRNA transfected, and CAT-2 siRNA transfected infected macrophages, respectively, in comparison to uninfected macrophages. Simultaneously, it was observed that knock down of CAT-1 had no significant effect on macrophage putrescine and spermidine level. However, CAT-2 knock down decreased the putrescine level by ~2.7-fold (Figure 9E) and spermidine level by ~1.9-fold (Figure 9F) in *Leishmania*-infected macrophages compared to control siRNA transfected infected macrophages. Therefore, our results showed clear decrease in the level of polyamines in infected macrophages in both l-arginine deprivation as well as during inhibition of l-arginine transport.

### Significance of Arginase–iNOS Expression in the Survival of *Leishmania* inside Macrophages

Arginase–iNOS expression critically regulates the outcome of infection. In this study, we wanted to explore the role of arginase and iNOS in the regulation of *Leishmania* infection. It was observed that arginase inhibition decreased the parasite load by ~3.8-fold, whereas, iNOS inhibition increased the parasite load by ~1.7-fold (Figure 10A). Similar observation was found in case of measurement of percent infectivity. Arginase inhibition led to a decreased percent infectivity by ~1.9-fold (Figure 10B).

**Figure 10:** Effect of regulation of arginase-inducible nitric oxide synthase (iNOS) balance in *Leishmania donovani* survival inside macrophages. THP-1 monocyte-derived MΦs were either left untreated or preincubated with BEC (200 µM) or L-NIL (100 ng/ml) for 3 h followed by infection with *L. donovani* for 48 h **(A,B,E,G,H)**. In another experiment, THP-1 MΦs were transfected with control siRNA, Arg-1, Arg-2, or iNOS siRNA followed by infection with *L. donovani* for 48 h **(C,D,F,I,J)**. Intracellular parasites were visualized by staining the cells with Giemsa followed by optical microscopy at 100× oil immersion. The parasite load was measured by counting the number of intracellular amastigotes per 100 macrophages **(A,C)**. The rate of infection was analyzed by counting the percent infected macrophages **(B,D)**. Extracellular nitrite level was measured by Griess method using NaNO_2_ as standard **(E,F)**. The polyamines (putrescine and spermidine) were extracted by TCA precipitation followed by dansyl chloride derivatization, separation by reverse-phase high performance liquid chromatography as described in “Materials and Methods.” Dansylated putrescine **(G,I)** and dansylated spermidine **(H,J)** were quantified by fluorescence spectrometry. Each experiment was repeated three times. Each determination was made in triplicate and the values were expressed as mean ± SD for three independent experiments. Kruskal–Wallis with Dunn’s multiple comparison test was used to evaluate statistical significance for comparing three or more groups; *p < 0.05; **p < 0.005; ns, non-significant.

RETRACTED

Parasite load and percent infectivity was further measured in Arg-1, Arg-2, and iNOS siRNA transfected and *Leishmania*-infected macrophages. It was observed that silencing of Arg-1 decreased the parasite load by ~3.3-fold (Figure 10C) and percent infectivity by ~1.9-fold (Figure 10D) in comparison to control siRNA transfected macrophages. On the other hand, silencing of Arg-2 decreased the parasite load by ~2.1-fold (Figure 10C) when compared to control siRNA transfected macrophages. However, in case of Arg-2 knock down percent infectivity was not significantly altered (Figure 10D). However, silencing of iNOS increased the parasite load by ~1.9-fold (Figure 10C). Therefore, our results indicated that arginase expression is critically involved in promoting parasite survival inside macrophages.

Simultaneously, inhibition of arginase activity by BEC also resulted in ~1.8-fold increased NO level in infected macrophages (Figure 10E). Silencing of macrophage Arg-1 and Arg-2 also increased the NO level in *Leishmania*-infected macrophages by ~1.8-fold and ~1.3–fold, respectively (Figure 10F).

Further, polyamines were also measured in *Leishmania*-infected macrophages pretreated with inhibitor of arginase and iNOS. It was observed that BEC pretreatment decreased the putrescine level by ~2.7-fold (Figure 10G) and spermidine level by ~1.9-fold (Figure 10H) in infected macrophages when compared to untreated infected macrophages. However, pretreatment of L-NIL increased the putrescine level by ~1.8-fold (Figure 10G) and spermidine level by ~1.6-fold (Figure 10H) in infected macrophages when compared to untreated infected macrophages. Polyamine level was also measured in Arg-1, Arg-2, and iNOS downregulated *Leishmania*-infected macrophages. Putrescine level was found to be decreased by ~3.7-fold and ~2.0-fold (Figure 10I) and spermidine level by ~1.8-fold and ~1.3-fold (Figure 10J), respectively, in Arg-1 and Arg-2 siRNA transfected *Leishmania*-infected macrophages. However, iNOS knock down increased the putrescine level by ~1.9-fold (Figure 10I) and spermidine level by ~2.2-fold (Figure 10J) in *Leishmania*-infected macrophages compared to control siRNA transfected infected macrophages. These findings possibly suggest that arginase and iNOS expression are reciprocally regulated in case of *Leishmania* infection and the balance between these two enzymes regulate production of NO and polyamines and thereby determines the fate of *Leishmania* survival inside macrophages.

RETRACTED

### l-Arginine Availability and Transport Regulates Host Th1/Th2 Cytokine Response in Infected Macrophages

The involvement of l-arginine transport in regulation of Th1/Th2 balance in *Leishmania* infection was assessed by measuring cytokines at the transcript level by semi-quantitive RT-PCR as well as quantitive real-time PCR and released level by sandwich ELISA. The expression of Th2 cytokine, IL-10 was increased by ~3.2-fold in *Leishmania*-infected macrophages when compared to uninfected macrophages in l-arginine-supplemented media (Figure 11A). Simultaneously, IL-10 expression in infected macrophages was found to be reduced significantly in l-arginine deprived condition when compared to l-arginine-supplemented condition (Figures 11A,B). However, l-arginine deprivation had no significant effect on Th1 cytokine production in infected macrophages (Figures 11A,B). Cytokine expressions were further measured in *Leishmania*-infected macrophages in presence or absence of NEM. IL-10 level was found to be decreased by ~4.6-fold in NEM pretreated infected macrophages when compared to untreated infected macrophages (Figure 11C). However, pretreatment of macrophage with NEM had no significant effect on IL-12 and TNF-α level in infected macrophages (Figures 11C,D). The expression of cytokines was further checked in CAT-1 and CAT-2 siRNA transfected *Leishmania*-infected macrophages. Silencing of CAT-1 decreased the IL-10 level by ~1.9-fold in infected macrophages. However, CAT-2 knock down decreased the IL-10 expression by ~2.8-fold in *Leishmania*-infected macrophages when compared to control siRNA transfected macrophages (Figure 11E). Moreover, CAT-2 knock down decreased the IL-12 level by ~1.3-fold and had no significant effect on expression of TNF-α in infected macrophages (Figure 11E). Our real-time PCR data further validate the results of semi-quantitive RT-PCR (Figure 11F).

**Figure 11:** l-Arginine availability and transport regulate expression of pro-inflammatory and anti-inflammatory cytokines in infected macrophages. THP-1 monocyte-derived MΦs (1 × 10^6^ cells/ml) were grown in l-arginine-supplemented and l-arginine-depleted RPMI medium followed by infection with *Leishmania donovani* (multiplicity of infection 1:10) for 48 h **(A,B)**. In a separate experiment, THP-1 MΦs (1 × 10^6^ cells/ml) were either left untreated or preincubated with 250 µM NEM for 10 min followed by infection with *L. donovani* for 48 h **(C,D)**. In another experiment, THP-1 MΦs (1 × 10^6^ cells/ml) were transfected with control siRNA, CAT-1, or CAT-2 siRNA followed by infection with *L. donovani* for 48 h **(E,F)**. The expression of IL-10, IL-12, and TNF-α were determined at the transcript level by semi-quantitative RT-PCR **(A,C,E)** and quantitative real-time PCR **(B,D,F)**. The intensity of the bands was quantified by densitometry in Quantity one software. Each experiment was repeated three times. Each determination was made in triplicate and the values were expressed as mean ± SD for three independent experiments. Semi-QRT PCR gel images are representative of three experiments. Densitometric plots are shown below the gel images. Kruskal–Wallis with Dunn’s multiple comparison test was used to evaluate statistical significance for comparing three or more groups; *p < 0.05; **p < 0.005; ns, non-significant.

RETRACTED

To further validate our semi-quantitative data, we measured the concentration of cytokines at the released level by sandwich ELISA. Th2 cytokine, IL-10 level was increased by ~2.1-fold in *Leishmania*-infected macrophages when compared to uninfected macrophages in normal condition (Figure 12A). However, when Th2 cytokine released by *Leishmania*-infected macrophages in l-arginine deprivation and l-arginine supplementation condition was compared, significant decrease in IL-10 level (~1.9-fold; *p* ≤ 0.005) was observed in case of l-arginine deprivation. Moreover, l-arginine deprivation had no significant effect on Th1 cytokine production in infected macrophages (Figure 12A). Cytokines were further measured in *Leishmania*-infected macrophages in presence or absence of NEM. It was observed that IL-10 level was decreased by ~1.9-fold in NEM pretreated infected macrophages compared to untreated infected macrophages (Figure 12B). However, pretreatment of macrophages with NEM had no significant effect on IL-12 and TNF-α level in infected macrophages.

**Figure 12:** l-Arginine availability and transport regulate release of pro-inflammatory and anti-inflammatory cytokines in *Leishmania*-infected macrophages. THP-1 monocyte-derived MΦs (1 × 10^6^ cells/ml) were grown in l-arginine-supplemented and l-arginine-depleted RPMI medium followed by infection with *Leishmania donovani* (multiplicity of infection 1:10) for 48 h **(A)**. In a separate experiment, THP-1 MΦs (1 × 10^6^ cells/ml) were either left untreated or preincubated with 250 µM NEM for 10 min followed by infection with *L. donovani* for 48 h **(B)**. In another experiment, THP-1 MΦs (1 × 10^6^ cells/ml) were transfected with control siRNA, CAT-1, or CAT-2 siRNA followed by infection with *L. donovani* for 48 h **(C)**. Level of IL-10, IL-12, and TNF-α in the macrophage culture supernatants were quantified by sandwich ELISA **(A–C)**. Each experiment was repeated three times. Each determination was made in triplicate and the values were expressed as mean ± SD for three independent experiments. Kruskal–Wallis with Dunn’s multiple comparison test was used to evaluate statistical significance for comparing three or more groups; *p < 0.05; **p < 0.005; ns, non-significant.

RETRACTED

The level of cytokines in CAT-1 and CAT-2 siRNA transfected *Leishmania*-infected macrophages was also measured. It was observed that silencing of CAT-1 had no significant effect on cytokine release in infected macrophages. CAT-2 silencing decreased the IL-10 level by ~2.0-fold in *Leishmania*-infected macrophages compared to control siRNA transfected macrophages (Figure 12C). However, CAT-2 knock down had no significant effect on release of IL-10 and TNF-α in infected macrophages (Figure 12C). These findings clearly indicate that *Leishmania* infection is characterized by significant increased level of IL-10 cytokine. Inhibition of l-arginine transport decreased IL-10 level resulting in decreased parasite survival inside macrophages.

## Discussion

Arginine is one of the metabolic and signaling molecule required for protein synthesis by macrophages and their growth (54). Macrophages require exogenous arginine to meet their metabolic demands and it is also the key amino acid which signals M1 and M2 activation (55, 56). It is documented that when *Leishmania* enters inside the macrophage, instead of being classically activated, macrophage becomes alternatively activated and this ultimately promotes *Leishmania* survival inside macrophages. Simultaneously, inside the phagolysosome, the parasite has to face relatively carbohydrate sparse environment and, therefore, possibly uptakes fatty acids and amino acids as alternate energy sources for their survival and other activities (57–59). In our previous report, we have shown that l-arginine is crucial for the survival of *L. donovani* promastigotes *in vitro* (43). However, the role of l-arginine in the intra-macrophage survival of *L. donovani* is yet not properly elucidated. In the present study, we have investigated how *L. donovani* utilizes host l-arginine metabolic pathway and survives inside macrophages. Our results showed that the parasite load and percent infectivity was significantly reduced upon removal of l-arginine from the culture medium indicating the importance of l-arginine for the survival of *L. donovani* inside macrophages. Similar observations were reported by Sans-Fons et al. who demonstrated that the availability of l-arginine critically regulates macrophage activation and thereby promoting susceptibility to *L. major* infection (60).

RETRACTED

Previously, Darlyuk et al. reported that starvation resulted in increase in l-arginine uptake in *Leishmania* promastigotes after amino acid depletion, along with concomitant increase of LdAAP3 at both mRNA and protein levels (61). In our previous study, we also observed that l-arginine deprivation led to its increased uptake in *Leishmania* promastigotes (43). Therefore, although the role of *Leishmania* l-arginine transporters for their survival was reported earlier (61), there are few reports regarding the involvement of macrophage l-arginine transporters for intracellular survival of *Leishmania*. Wanasen et al. previously reported the involvement of mouse cationic amino acid transporter 2B (mCAT-2B) in case of *L. braziliensis* infection (62). Later, Sans-Fons et al. also reported that the growth enhancement of *L. major* amastigotes inside macrophages was associated with CAT-2-mediated l-arginine transport (60). In this study, we also observed that the expression of CAT-2 is specifically increased in case of *L. donovani* infection. CAT-2 level was found to be further increased upon l-arginine deprivation during *Leishmania* infection. Therefore, we hypothesized that upon sensing low l-arginine availability, *L. donovani* modulates the expression of macrophage l-arginine transporters particularly CAT-2 and increases the uptake of l-arginine for its survival and growth. However, as we observed that even in case of knock down of CAT-2, macrophage l-arginine transport is not decreased in normal condition, it is evident that l-arginine is transported by CAT-1 transporter in normal resting condition. Simultaneously, from the parasite load and percent infectivity data in case of CAT-1 and CAT-2 downregulation, we observed that CAT-2 downregulation had more pronounced effect than CAT-1 in decreasing parasite survival inside macrophages. Therefore, we hypothesize that when the amount of l-arginine required by *Leishmania* for intra-macrophage survival is not sufficient by CAT-1 mediated transport, then the parasite upregulates host CAT-2 expression, and utilizes CAT-2 mediated l-arginine supply. Further, we observed that when l-arginine transporters were blocked either by inhibitor or siRNA treatment, *L. donovani* survival was greatly reduced indicating the importance of l-arginine transport for their survival inside macrophages. Therefore, our results are in agreement with the study of Wanasen et al (62).

RETRACTED

Previous studies have demonstrated that pathogens take up extracellular l-arginine and compete with iNOS for l-arginine substrate to evade host defense (63). In this study, we observed that deprivation of l-arginine did not impair the upregulation of macrophage iNOS and arginase in normal condition. Similar results were reported in peritoneal exudate MΦ by Choi et al., where they have shown that MΦ activation and biological functions are not altered by the lack of l-arginine (64). However, our results are in contrary to the findings of El-Gayar et al. who showed that the presence of arginine is requisite for adequate translation of iNOS (65). In this study, we observed that host arginase is induced upon *Leishmania* infection and its expression is regulated by l-arginine availability in extracellular milieu and upon expression of CAT-2. Our study is the first to report that l-arginine transport is a critical factor for *L. donovani* infection *ex vivo* and this transport differentially regulate the expression of arginase in infected macrophages. However, as we observed that even in case of knock down of CAT-1, the expression of Arg-1 was decreased at the transcript level, we assume that CAT-1 mediated l-arginine transport might also have a role in regulation of arginase activity in *L. donovani*-infected macrophages. Our observation indicates that induction of host arginase is important for the survival of *L. donovani* parasite inside macrophages. In contrary to our observation, Wanasen et al. described that the l-arginine dependent intra-macrophage *L. amazonensis* survival was independent of arginase–iNOS activities (62). However, our findings is correlated with the studies by Boitz et al. who have recently shown that leishmanial arginase is not essential for proliferation of intracellular amastigotes, indicating that the parasites utilize host arginase pathway for their survival inside macrophages (34).

The conversion of l-arginine to l-ornithine and urea and its participation in polyamine production has been reported to stimulate growth of many pathogens, including *Leishmania* spp. (18, 26)., *Trypanosoma* spp. (20)., *Helicobacter pylori* (66) and *Mycobacterium bovis* (67). Several organisms, including *Leishmania* spp., can both synthesize polyamines *de novo* and salvage them by transport across their plasma membranes. In the present study, we observed that polyamine production was greatly diminished due to l-arginine deprivation or blockade of l-arginine transport ultimately resulting in decreased parasite survival inside macrophages.

RETRACTED

The metabolism of arginine by iNOS or arginase 1 produces radically different biological products (68). It is reported that iNOS generates NO in large quantities and under physiological conditions plays an important role in killing parasites (69) whereas arginase 1 in turn regulates NO through depletion of arginine availability (68). In the present study, we wanted to understand how the expressions of iNOS and/or arginase are regulated in macrophages after *L. donovani* infection. We observed that iNOS and arginase are reciprocally regulated. If arginase is inhibited, iNOS expression is increased resulting in increased production of NO. In contrast, if iNOS is inhibited, arginase activity got increased favoring *Leishmania* survival inside macrophages. Elevated arginase activity has also been documented by multiple investigators in animal models of cancer (70, 71) and recently in human (72, 73). Thus, it is possible that increased arginase 1 expression may downregulate the production of NO as it limits arginine accessibility for iNOS. The present study for the first time revealed that l-arginine transport is a crucial factor for *L. donovani* infection *ex vivo* and that this transport system could moderately explain the differential expression of arginase and iNOS in infected macrophages. Our experiments point to a link between reduced l-arginine transport and decreased *L. donovani* growth. The data presented here provide a new explanation for the intracellular parasite replication in *L. donovani* infections.

The catabolism of l-arginine by macrophages plays a crucial role in regulation of the immune response, in several parasitic diseases including *L. major* infection (74). It is reported that to evade immune responses, some pathogens induce arginase expression in the host (75, 76) and that high level of arginase production blocks the immune response by local depletion of l-arginine (77). In this study, we investigated the involvement of l-arginine transport in regulation of Th1/Th2 balance in *L*. donovani infection. Our findings clearly indicated that *Leishmania* infection is associated with increase in IL-10 level and inhibition of l-arginine transport significantly decreased IL-10 level resulting in decreased parasite survival inside macrophages. Our findings are in agreement with the studies of Hesse et al. (56). Therefore, we propose that the IL-10 released by the macrophages in case of l-arginine availability in extracellular milieu induce the host arginase pathway leading to polyamine production and thereby promoting *L. donovani* survival inside macrophages.

RETRACTED

In conclusion, our results decipher that l-arginine availability and transport plays a crucial regulatory role for survival of *L. donovani* parasite inside macrophages. *L. donovani* upregulates host l-arginine transport and controls l-arginine metabolism resulting in increased production of polyamines and skewed immune response for their survival inside macrophages (Figure 13). Our study is the first report describing the importance of CAT-2 mediated l-arginine transport for survival of *L. donovani* inside macrophages. The findings presented here further increase our knowledge about the pathways by which l-arginine deprivation regulates host immune response and promotes *Leishmania* survival inside macrophages. Therefore, targeting the metabolism of l-arginine and the macrophage cells expressing l-arginine-metabolizing enzymes is likely to constitute an important therapeutic and prophylactic approach to treat VL.

**Figure 13:** Schematic representation demonstrating the role of l-arginine availability and transport in the modulation of host immune response and *Leishmania* survival inside macrophages. The model illustrates that the fate of *Leishmania* parasites inside macrophages depend on the availability of extracellular l-arginine and activation status of macrophages. If l-arginine is available, it is taken up from the external medium by cationic amino acid transporters (CAT-2) and metabolized by arginase and other polyamine biosynthetic and thiol metabolic pathway enzymes, such as ornithine decarboxylase (ODC), spermidine synthase (SpdS), spermine synthase (Sps) to produce l-ornithine, putrescine, spermidine, and spermine. *Leishmania* acquires either arginine or polyamines by the transporters present on the membrane of the parasitophorous vacuole which promotes amastigote proliferation and cell growth. Simultaneously, l-arginine can also be utilized by inducible nitric oxide synthase (iNOS) to produce nitric oxide (NO) that would kill *Leishmania* parasites. *Leishmania* infection modulate the host to downregulate this pathway for their survival.

## Ethics Statement

This study was carried out in accordance with the recommendations of Institutional Human Ethical Committee of the Rajendra Memorial Research Institute of Medical Sciences (Patna, India) with written informed consent from all subjects. All subjects gave written informed consent in accordance with the Declaration of Helsinki. The protocol was approved by the Institutional Human Ethical Committee of the Rajendra Memorial Research Institute of Medical Sciences (Patna, India).

## Author Contributions

Conceived and designed the experiments: AM, SD, and PD. Performed the experiments: AM, AjayK, SR, SV, AG, SS, RS, and KA. Analyzed the data: AM, SD, AG, CM, and PD. Contributed reagents/materials/analysis tools: SR, AS, BP, AshishK, CM, and PD. Wrote the paper: AM, SD, and PD.

RETRACTED

## Conflict of Interest Statement

The authors declare that the research was conducted in the absence of any commercial or financial relationships that could be construed as a potential conflict of interest.
